The article "MicroRNA modulators of epigenetic regulation, the tumor microenvironment and the immune system in lung cancer" was published in 2015. Journal: Mol Cancer.

# MicroRNA modulators of epigenetic regulation, the tumor microenvironment and the immune system in lung cancer

**DOI:** 10.1186/s12943-015-0302-8

**Published:** 2015-02-07

**Authors:** Anna Maria Rusek, Mohammed Abba, Andrzej Eljaszewicz, Marcin Moniuszko, Jacek Niklinski, Heike Allgayer

**Affiliations:** Department of Clinical Molecular Biology, Medical University of Bialystok, Waszyngtona 13, Białystok, 15-269 Poland; Department of Experimental Surgery, Medical Faculty Mannheim, Heidelberg University, Theodor Kutzer Ufer 1-3, 68135 Mannheim, Germany; Molecular Oncology of Solid Tumors, DKFZ (German Cancer Research Centre), Im Neuenheimer Feld 280, 69120 Heidelberg, Germany; Department of Regenerative Medicine and Immune Regulation, Medical University of Bialystok, Bialystok, Waszyngtona 13, Białystok, 15-269 Poland

**Keywords:** microRNA, Lung cancer, Epigenetic regulation, Tumor microenvironment

## Abstract

Cancer is an exceedingly complex disease that is orchestrated and driven by a combination of multiple aberrantly regulated processes. The nature and depth of involvement of individual events vary between cancer types, and in lung cancer, the deregulation of the epigenetic machinery, the tumor microenvironment and the immune system appear to be especially relevant. The contribution of microRNAs to carcinogenesis and cancer progression is well established with many reports and investigations describing the involvement of microRNAs in lung cancer, however most of these studies have concentrated on single microRNA-target relations and have not adequately addressed the complexity of their interactions. In this review, we focus, in part, on the role of microRNAs in the epigenetic regulation of lung cancer where they act as active molecules modulating enzymes that take part in methylation-mediated silencing and chromatin remodeling. Additionally, we highlight their contribution in controlling and modulating the tumor microenvironment and finally, we describe their role in the critical alteration of essential molecules that influence the immune system in lung cancer development and progression.

## Introduction

One of the most promising molecular entities to have impacted cancer research in recent times is the group of small non-coding RNAs known as microRNAs. Since the first miRNA gene called lin-4 was discovered in *Caenorhabditis elegans* [1], several others have been identified, and so far over 2500 miRs have been described in the human genome miRBase (www.mirbase.org) [2]. MicroRNAs have been described to be involved in several cellular processes including proliferation, development, metabolism, differentiation and apoptosis. Importantly, the deregulation of microRNA expression and function has been linked to many human pathological conditions, including cancer [3,4].

Classically, in cancer, microRNAs have been categorized as either oncogenic or tumor suppressor miRNAs. In the first instance, by post-transcriptionally lowering mRNA and subsequently protein levels of molecules with tumor suppressor functions, microRNAs assume an oncogenic function. Conversely, by targeting oncogenic molecules, they act as tumor suppressors and the altered expression levels of the microRNA(s) between tumor and normal states coupled with the function of the targeted molecule(s) dictate the resulting (end) phenotype. Beyond the classical regulation of oncogenes and tumor suppressor mRNAs, aberrantly expressed microRNAs could in further levels of complexity act: 1) to regulate the epigenetic machinery by a) directly modulating enzymes which take part in methylation-mediated silencing and chromatin remodeling [5] or b) be epigenetically regulated themselves [6]; 2) in a paracrine fashion via exosomes, microvesicles and protein complexes to influence the tumor microenvironment [7-10] and 3) to promote the release of mediators which activate pro- or anti-cancer immune activity [11,12]. These latter mechanisms of microRNA regulation are explained in detail.

## MicroRNAs and epigenetic regulation in cancer

The epigenome is both dynamic and highly regulated in order to conserve normal expression patterns in cells. One of the most important components of expression regulation is the methylation of CpG islands within promoter regions both in normal as well as cancer cells [13,14]. The dynamic balance is maintained by a family of DNA methyltransferases: notably DNMT1 (maintenance DNMT) and DNMT3a and 3b (*de novo* DNMTs). Equally important in epigenetic regulation are covalent changes in histone tails that are orchestrated by histone methyltransferases (HMT), histone acetyltransferases (HAT), histone deacetylases (HDAC) [13,15] and polycomb proteins such as PRC 1 and PRC 2 [16]. MicroRNAs as a part of regulatory networks serve as significant targets for the epigenetic machinery and are also active players in modulating enzymes which take part in methylation mediated silencing and the chromatin remodeling machinery. MiR-127 was the first epigenetically regulated microRNA to be reported in a cancer entity [17]. Since then, many microRNAs were found to undergo epigenetic regulation in different cancer types including colorectal [18,19], urological [20], breast [21], ovarian [22,23], gastric [24] and pancreatic [25] as well as different types of haematological malignancies [26]. Most of the microRNAs are involved in crucial processes in the cell, thus, a great number of epigenetically regulated microRNAs (app. 45%) are implicated in several cancer types (eg., miR −124, −129, −34b at least 7 types, 34a −12 types), however, none of these have so far been found to be particularly involved in lung cancer [27].

### MicroRNAs regulated by methylation

Hypermethylation is one of the most common epigenetic regulatory mechanisms and about half of the microRNA genes are subject to hypermethylation of CpG regions of their promoters [6], resulting in microRNA silencing or down-regulation. There is ample evidence supporting this mode of action, for instance, CpG island hypermethylation mediated silencing of miR-124a has been found in a wide range of lung cancer cell lines, including H358, CALU3, A549, A427, H2126 and H209. Interestingly, the epigenetic loss of microRNA-124a was functionally related to an activation of cyclin D kinase 6 (CDK6) and an inactivating phosphorylation of the retinoblastoma tumor suppressor protein (pRb) [28]. A similar type of regulation was also observed with miR-199a silencing in several cancer cell lines that occurred as a result of gene methylation [29]. This microRNA negatively regulates the proto-oncogene c-Met and its downstream effector ERK2, thus the hypermethylation of its promoter acts as an oncogenic switch. Moreover, transfection of miR-199a into cancer cells increases their pro-apoptotic ability, suggesting that miR-199a can be a potential therapeutic molecule. Ceppi and colleagues discovered that methylation mediated down-regulation of miR-200c correlated with a higher invasive potential of NSCLC cell lines [30] with additional experiments showing inhibition of *in vitro* invasion and *in vivo* metastasis. Accordingly, miR-200c mimics restored sensitivity to therapeutic compounds such as Cisplatin and Cetuximab. Invariably, an association between low miR-200c expression, poor grade differentiation, a higher degree of lymph node affectation and a lower endogenous E-cadherin expression was observed in a patient cohort. MiR-200c is an important EMT mediator where it suppresses EMT by down-regulating ZEB proteins. ZEB1 and ZEB2 proteins are also targets for miR-141 and miR-429, which have also been shown to be hypermethylated in lung cancer [31]. In a study by Heller et al. [32], miR-9-3 and miR-193a were found to be tumor-specifically methylated in NSCLC patients. Moreover, patients with miR-9-3 methylated NSCLC had a significantly shorter disease-free survival and shorter overall survival than the unmethylated control group. This data supports the idea, that miR-9-3 methylation could be an interesting prognostic parameter in patients with NSCLC. In two independent studies, Wang and colleagues [33] and Watanabe and colleagues [34] showed that promoter hypermethylation mediated silencing of the miR-34b/c is a common event in NSCLC. Additionally, Wang et al. showed a strong association between aberrant methylation of the miR-34b/c gene and a high probability of relapse, poor overall survival and disease-free survival in patients with lung cancer. Furthermore, Watanabe’s study revealed that miR-34b/c expression negatively correlated with the expression of c-Met. Similarly, they also showed that the tumor suppressor activity of miR-126 that inhibits invasion by directly targeting Crk is silenced in lung cancer cells by the DNA methylation of its host gene, EGFL7. Interestingly, it was also shown that the promoter methylation status of the miR-503 gene may influence sensitivity of NSCLC cells to cisplatin, suggesting that epigenetic interference might be a promising way to improve existing therapies [35].

Taken together, the hypermethylation of microRNA genes or promoter sequences is an important mechanism leading to the down-regulation of microRNA expression resulting in a reversal of oncogene suppression (c-Met, CDK6, Crk), repression of tumor suppressor genes (pRB), or activation of proteins involved in epithelial-to-mesenchymal transition (EMT) (ZEB1/2). However, the converse is also true, for instance, the high expression of miR-196a in lung cancer samples and cell lines was attributed to DNA demethylation [36]. Moreover, miR-196a up-regulation correlated with a more advanced clinical stage and lymph node metastasis in lung cancer. *In vitro* functional experiments demonstrated that higher miR-196a expression levels promote cell proliferation, migration and invasion by targeting and suppressing the homeobox protein -A5 (HOXA5) at the protein as well as at the mRNA level. An inverse relation was then demonstrated in NSCLC tissues.

### MicroRNAs regulated by histone modifications

Aside methylation changes, histone modifications have also been implicated in the regulation of microRNA expression. Incoronato and colleagues [37] investigated the mechanism behind miR-212 silencing in lung cancer and by comparing Calu-1 (lung cancer cell line) and MRC5 (human fibroblasts), they found significant differences in the methylation status of H3K27 and H3K9 marks and in the acetylation status of H3K9, suggesting that modifications of histones on the miR-212 gene predicted transcriptional start sites contributing to its strong down-regulation in lung cancer. Additionally, an analysis of human tissue specimens of normal tissue and lung cancer revealed a correlation between miR-212 silencing and up-regulation of anti-apoptotic protein PED. Similarly, miR-373 silencing in lung cancer was found to be deacetylase-dependent with consequences on cell proliferation, migration, invasion and the expression of mesenchymal markers that appear to be modulated through IRAK2 and LAMP1 [38].

Interestingly, instances exist where certain microRNAs that have been established as key players in several cancer types including lung cancer [39], have been found to be regulated by epigenetic mechanisms in some of these tumor entities, but not in lung cancer. This is the case with miR-155, which in addition to being one of the most consistently regulated microRNAs in lung cancer, has equally significant prognostic significance [40,41]. Whereas miR-155 was found to be repressed by deacetylation of H2A and H3 through a mechanism mediated by BRCA1 in breast cancer [42], such reports are lacking in lung cancer, even though BRCA1 is not that unimportant in lung cancer [43].

### MicroRNAs regulating the epigenetic machinery – Epi-microRNAs

MicroRNAs can also act as modifiers of the epigenetic network. These so-called epi-microRNAs contribute to altered epigenomic patterns in cancer cells, with the first evidence of such microRNA activity observed in lung cancer cell lines, where the miR-29 family (29a, 29b and 29c) was found to directly target the *de novo* DNA methyltransferases, DNMT-3a and DNMT-3b, inhibiting their activity. Consequently, this action resulted in a re-activation of silenced tumor suppressor genes (FHIT, WHOX), thus preventing tumor progression [5]. However, in contrast to the large number of studies conducted in different cancer types, very few reports exist on microRNAs that regulate the epigenome in lung cancer. Of the studies documented in lung cancer, was one where Xi et al. reported that the repression of miR-487b in cultured cells exposed to cigarette smoke, and in primary lung cancers correlated with an overexpression of the polycomb repressor proteins BMI1 and SUZ12 [44]. Interestingly, this state coincided with miR-487b gene methylation and *de novo* nucleosome occupancy in its area, indicating that the microRNA also epigenetically regulated itself. Besides its function of epigenetic regulation, miR-487b also directly targets WNT5A, KRAS and MYC, suggesting a multiple mode of action. Another exciting example of the regulatory role of microRNAs in lung cancer epigenetics involves miR-449 [45]. This study showed that the down-regulation of miR-449 might be responsible for an overexpression of HDAC1, subsequently inhibiting cell growth and promoting tumor suppression. Similar work by Jeon and colleagues also revealed a therapeutic potential for miR-449, showing that co-treatment with miR-449 and a HDAC1 inhibitor led to significantly higher growth reduction than with the HDAC1 inhibitor itself. Further examples demonstrating this regulatory principle include the work done by Cho and colleagues [46] where they showed that the down-regulation of miR-101 affected enhancer of zeste homolog 2 (EZH2), a member of the polycomb repressive complex causing its overexpression. EZH2 is known to be involved in the methylation of H3K27, bringing about gene silencing and in the process regulating several cancer-associated processes. They found that the general methylation status of H3K27 was significantly higher in metastatic lung cancer than in primary lung cancer tissue, with in vitro studies showing a significant impact on invasion. Furthermore, EZH2 was also shown to be a direct target of miR-138 [47] where experiments on several lung cancer cell lines, as well as tissue samples from patients with NSCLC revealed that the down-regulation of miR-138 resulted in an up-regulation of EZH2 inhibiting apoptosis, G0/G1 cell cycle arrest and promoting cell proliferation and tumor invasion. A summary of microRNAs involved in epigenetic regulation are presented in Table 1.

**Table 1:** **MicroRNAs involved in epigenetic regulatory mechanisms in lung cancer**

**MicroRNA**	**Chromosome**	**Type of regulation**	**Target**	**Functional consequence**	**References**
**miR-124a-1**	8	Hypermethylation mediated silencing	CDK6	Oncogene activation, repression of tumor suppression	Lujambio et al., 2007 [28]
**miR-124a-2**	8		pRb		
**miR-124a-3**	20				
**mir-199a-1**	19	Hypermethylation mediated silencing	c-Met	Anti-apoptotic function	Kim et al., 2008 [29]
**mir-199a-2**	1		(ERK2)	Oncogene activation	
**miR-200c**	12	Hypermethylation mediated down-regulation	ZEB1	Promotion of EMT and metastasis	Ceppi et al., 2010 [30]
**miR-141**	12	Hypermethylation	ZEB1/2		Lopez Serra; Esteller, 2012 [31]
**miR-429**	1	Hypermethylation	ZEB1/2		Lopez Serra; Esteller 2012 [31]
**miR-9-3**	15	Methylation mediated down-regulation			Heller et al., 2012 [32]
**miR-193a**	17	Methylation mediated down-regulation		Altered expression regulation of genes involved in Proliferation, apoptosis, differentiation and adhesion	Heller et al., 2012 [32]
**miR-34b/c**	11	Promoter hypermethylation mediated silencing	(c-Met)	Oncogene activation, metastasis formation	Wang et al., 2011 [33]
					Watanabe et al., 2011 [34]
**miR-503**	X	Promoter methylation mediated silencing	FANCA	Modulate sensitivity to cisplatin regulate apoptosis	Li et al., 2014[35]
**miR-126**	9	Host gene promoter methylation mediated silencing	Crk	Oncogene activation	Watanabe et al., 2011 [34]
**miR-196a-1**	17	Demethylation mediated up-regulation	HOXA5	Promotion of cell proliferation, migration and invasion.	Liu Xiang-hua et al., 2012 [36]
**miR-196a-2**	12				
**miR-212**	17	Histone tail methylation mediated down-regulation	PED	Anti-apoptotic function	Incoronato et al., 2011 [37]
**miR-373**	19	Histone acetylation mediated silencing	IRAK2	Promotion of cell proliferation, migration, and invasion, Pro-EMT function	Seol et al., 2014 [38]
			LAMP1		
**miR-29a**	7	MicroRNA’s downregulation mediates DNMT	DNMT3a	Repression of tumor suppression	Fabbri et al., 2007 [5]
**miR-29b-1**	7	Up-regulation	DNMT3b		
**miR-29b-2**	1		(FHIT		
**miR-29c**	1		WHOX)		
**miR-487b**	14	MicroRNA’s repression mediates target Genes overexpression	*SUZ12*, *BMI1*, *WNT5A*, *MYC*, *K-ras*	Promotion of tumor progression and metastasis	Xi et al.,2013 [44]
**miR-449**	5	MicroRNA’s down-regulation mediates HDAC1	HDAC1	Repression of tumor suppression	Jeon et al., 2011 [45]
		Up-regulation		Promotion of tumor metastasis	
**miR-101-1**	1	MicroRNA’s down-regulation mediates EZH2	EZH2	Promotion of EMT and tumor metastasis	Cho et al., 2011 [46]
**miR-101-2**	9	Up-regulation	(CDH1, MMP-2)		
**miR-138-1**	3	MicroRNA’s down-regulation mediates EZH2	EZH2	Promotion of proliferation, repression of apoptosis, Disruption of cell cycle arrest	Zhang et al., 2013 [47]
**miR-138-2**	16	Up-regulation			

A compilation of the most significant microRNAs targeted by epigenetic regulatory mechanisms, including those that modulate epigenetic changes in lung cancer. The most important functional outcomes are described. Genes placed in brackets are not targeted directly.

## MicroRNAs and the tumor microenvironment

The tumor microenvironment is an increasingly appreciated item of interest in cancer development and progression. During cancer progression, sequences of molecular changes arise in the tumor as well as in the neighboring tissue stroma. Since tumor development is driven by physiological responses to an aberrant stromal environment [48] the interaction between the tumor and stromal cells determines the outcome of progression [49]. The tumor microenvironment is a complex structure that in addition to the extracellular matrix (ECM) comprises many other cell types, including endothelial cells, inflammatory cells and most abundantly, fibroblasts [50] While normal fibroblasts have been found to prevent tumor progression [51] the so-called cancer associated fibroblasts (CAFs) generate an environment promoting tumor growth and invasiveness [52]. CAFs are characterized by specific changes in their secretory profile, e.g, chemokines that attract inflammatory cells. Together, they release growth factors that trigger cancer cell proliferation, inhibit apoptosis or indirectly stimulate angiogenesis [53]. Interestingly, one of the major mechanisms by which CAFs are activated is mediated by specific microRNAs, e.g. miR-21, miR-31, −214, and 155 [7,8]. There is ample evidence, that microRNAs are not only present in the cells, but also in extracellular space [54,55]. Importantly, extracellular microRNAs also play a very vital role in cell to cell communication [9] and are capable of contributing to microenvironment-associated processes such as angiogenesis, matrix degradation and stromal remodeling, all which support cancer progression and metastasis [10]. About 90% of microRNAs found in the ECM are bound to RNA- binding proteins (eg. AGO proteins, especially Ago2, NPM1 - nucleoplasmin 1 and GW 182 responsible for microRNA stabilization as well as secretion) and just 10% exist in extracellular vesicles such as exosomes, apoptotic bodies and, mainly microvesicles (MVs) [9,55,56]. Remarkably, most of the microRNAs that are differentially expressed in CAFs are down-regulated as compared with normal fibroblasts, suggesting that they act as suppressors of stromal activation [57]. Evidence for the contribution of microRNAs in lung cancer angiogenesis arising from a specific influence on the tumor microenvironment was hinted at in the study by Jusufovic and colleagues [58] who found significantly higher microvessel density (MVD) together with decreased expression levels of let-7b and miR-126 in tumor and surrounding tissue of 50 NSCLC patients as compared to corresponding normal tissues. Interestingly, there was no difference in expression between tumor and surrounding tissue for both microRNAs and MVD, indicating similar molecular changes in the tumor and surrounding cells in this context [58].

In addition to influencing the local microenvironment, tumor cells have also been shown to secrete exosomes at a significantly higher level compared to normal cells [59]. These so-called tumor-derived exosomes (TD exosomes) contain pro-tumorigenic components, in particular abundant microRNAs which influence and modify stromal cells and recruit them as cancer-associated stromal cells, which in turn influence cancer cells and the ECM contributing to cancer development and progression [10,59]. Additionally, a mechanism based on passive leakage has been proposed, in which microRNAs are released from the cells due to injury, chronic inflammation, necrosis, or from cells with very short half-lives, like platelets [60].

Notable instances of microRNA regulation of the tumor microenvironment in lung cancer include the repression of the angiogenic program by IL-8, ICAM and CXCL1 through the lung tumor cell mediated exosomal release of miR-192 with a consequent reduction in metastatic burden and tumor colonization [61]. In another study, TGF-β induced release of miR-183 by lung cancer cells was found to control DAP12, a critical stimulatory signal adaptor linked to numerous NKC receptors resulting in a suppression of NK cell function [62]. Still, Krysan and colleagues found the inflammatory molecule, prostaglandin E2 (PGE2) to mediate an up regulation of c-Myc in stromal cells, which in turn modulates the expression of the miR-17-92 cluster, that effectively targets the tumor suppressor PTEN. The end effect was an augmentation of apoptosis resistance in non-small cell lung cancer (NSCLC) cells [63]. In what appears to be an interesting example of the microenvironment of one organ affecting the dissemination of cells from a different organ, Subramani et al., found that miR-768-3p released by brain astrocytes targets K-ras, mitigating metastatic potential of lung cancer cells. The down-regulation of this microRNA seen in many brain tumors is thought to enhance K-ras expression, including its downstream effectors ERK1/2 and B-Raf, and thus promoting metastasis [64].

## MicroRNAs and immune responses in lung cancer

In addition to the processes described above, it has become increasingly clear that microRNAs play multiple roles in the negative regulation of numerous immune responses triggered by rapidly proliferating neoplastic cells. The genetic instability of neoplastic cells is associated with alterations of antigenic patterns that may in turn lead to attenuated recognition of the tumor by immune cells [65]. Some of these alterations are largely influenced by actions mediated by a constellation of different microRNAs (Figure 1). An example of this is miR-9 that is over-expressed in many cancers including lung cancer [66]. MiR-9 is capable of down-regulating the transcription of the MHC class I gene, thereby preventing the recognition of tumor cells by the immune system [11,56]. On the other hand, a down-regulation of miR-29 expression in cancer leads to an up-regulation of B7-H3 gene transcription and the subsequent expression of this molecule on the surface of neoplastic cells [67]. Consequently, *B7-H3* delivers an inhibitory signal to T cells and NK cells and therefore inhibits the anti-tumor activity mediated by these cells [68,69]. Similarly, miR-222 and −339 down-regulate the expression of intracellular cell adhesion molecule 1 (ICAM-1) on the surface of tumor cells [70]. The binding of ICAM - to lymphocyte function-associated antigen (LFA-1) has been shown to be essential for optimal activation of cytotoxic T cell (CTLs) [71], thus, miR-222 and −339 in cancer cells contribute to impaired CTL-mediated tumor cell lysis [70]. Moreover miRs-221 and −222 are overexpressed in NSCLC and act in part by targeting TIMP3 [72] which has known functions in controlling cytokine and growth factor homeostasis. Furthermore, several microRNAs, for instance miRs-21 and −126/126*, contribute to the modulation of the tumor microenvironment, which encompasses not only stroma cells but also soluble factors and signaling molecules [73-76] (Figure 1). Regulatory T lymphocytes (Tregs), are important components of the tumor stroma, and are known to predominantly exert immunosuppressive effects. A number of tumor-bound chemokines including CCL22 have been shown to recruit Tregs to modulate immune responses in cancer [77]. Notably, CCL22 production in cancer cells is regulated by miR-34a, which suppresses the expression of this chemokine. On the other hand, increased levels of TGF-β in the tumor milieu down-regulate the expression of miR-34a and thereby increase infiltration of immunosuppressive Tregs. The TGF-β - miR-34a - CCL22 axis is therefore important in modulating the tumor microenvironment [78]. Other chemokines such as CXCL12 (Sdf-1) and CCL2 (MCP-1) are secreted by various cancer types and function as autocrine growth factors as well as chemo-attractants for progenitor cells and monocytes/macrophages [12,79,80]. Interestingly, the transcription of the CXCL12 gene is controlled by miR126/miR126*. This microRNA pair directly inhibits the expression of CXCL12 and down-regulates the production of CCL2 in a CXCL12-dependent process in which stromal cells (mainly mesenchymal stem cells, MSCs) seem to play the crucial role. In cancer cells, decreased miR-126/126* expression results in an increased production and secretion of CXCL12 that in turn attracts MSCs to the tumor microenvironment and increases the secretion of CCL2 [75]. Subsequently, CCL2 recruits monocytes/macrophages to the site of neoplastic growth [81].

**Figure 1:** **MicroRNA-mediated regulation of tumor microenvironment.** The scheme demonstrates involvement of microRNAs in chemokine-mediated recruitment of regulatory T cells, monocytes, macrophages and MSCs and the role of microRNAs in tumor-related dysfunction of NK and cytotoxic T cells. All microRNAs are shown in red while gene targets and types of responses are shown in black. Arrows indicate directions of cause-and-effect relationships.

During migration, monocytes are exposed to many signals derived from cancer and stromal cells that induce their differentiation towards classically (M1) or alternatively activated (M2) macrophages. Tumor associated macrophages (TAMs) control the majority of immunological processes within tumors exerting both, regressive (M1) or progressive (M2) effects on the tumor development [82,83]. Unfortunately, the vast majority of TAMs exhibit an M2-like phenotype. Remarkably, a significant number of microRNAs like miRs-9, −21 and −146 are involved in the differentiation of the TAMs from peripheral blood monocytes (Figure 2). Both monocytes/macrophages and cancer cells are capable of releasing different pro- and anti-inflammatory cytokines like the immunosuppressive cytokine IL-10, which fosters tumor growth [84]. Substantial amounts of this cytokine are secreted by neoplastic cells including that of the lung [85,86]. Interestingly, the transcription of the IL-10 gene in tumor cells is indirectly regulated by miR-30d, which acts by directly repressing GALNT7. GALNT7 suppression leads to increased production and secretion of IL-10, which in turn promotes monocyte differentiation towards the M2 phenotype [87]. In addition, in human monocytes, IL-10 up-regulates miR-187 expression which down-regulates TNF-α production. Moreover, in macrophages, miR-187 indirectly decreases the expression of IL-6 and IL-12p40 via decreasing MAIL in an NFKBIZ-dependent manner [88]. Along similar lines, the differentiation of monocytes towards M2 macrophages can be induced by M-CSF. M-CSF signaling down-regulates miR-142-3p in monocytes which leads to increased Egr2 (Krox20) expression. This transcription factor can control differentiation of monocytes via activating macrophage-specific genes such as C-FMS, acting in cooperation with Spi-1/PU.1 [89].

**Figure 2:** **MicroRNA-mediated control of monocyte differentiation and tumor associated macrophages (TAMs) functions.** All microRNAs are shown in red while gene targets and types of responses are shown in black. Arrows indicate directions of cause-and-effect relationships.

Many of the pro-tumorigenic outcomes of TAMs’ are controlled by microRNAs and depend on such factors like HMGB1 and IL-10 [88,90]. These mediators are secreted both by tumor cells and stroma and act via interactions with several cell surface receptors including toll-like receptors (TLR) and the IL-10 receptor. TLR2-, TLR-4- and TLR5-mediated signaling and NF-κβ activation in macrophages up-regulates the expression of miR-146 that in turn targets IRAK1 and TRAF6, proteins which are crucial components of interleukin-1- and TNF-related signaling pathways, respectively. More specifically, miR-146 acts via targeting IRAK1 and TRAF6, members of the TLR-NF-κβ pathway, and therefore contributes to controlling the expression of an array of inflammatory cytokine genes. MiR-146 therefore acts through a negative feedback loop and down-regulates cytokine signaling [91]. On another note, miR-92 is up-regulated following TLR-4 activation and in turn down-regulates the expression of TNF-α and IL-6 [92]. TLR4-mediated up-regulation of miR-21 suppresses programmed cell death protein-4 (PDCD4) expression. This mechanism may limit pro-inflammatory cytokine production in macrophages via suppressing NF-κβ activation, leading to an increased IL-10 production [90]. Notably, miR-21 and miR-29a are expressed at different levels in various cancers including lung cancer [93-95]. Both miR-21 and miR29a can act within cancer cells or can be delivered from cancer cells to macrophages by microvesicles and can subsequently bind intracellular TLR7 or TLR8. This microRNA-TLR interaction leads to the activation of the NF-κβ pathway and an increase in the production of the pro-inflammatory cytokines, IL-6 and TNF-α that in turn activate pro-metastatic responses in TAMs [96]. Some microRNAs also mediate a cross talk between cancer and stromal cells as in the case of TAM-derived miR-223, which down-regulates Mef2c expression in neoplastic cells, leading to an increase of cancer cell invasion, probably through the involvement of the miR-223 – Mef2c – β-catenin pathway [97].

Taken together, substantial evidence supports the dynamic role of microRNAs within the tumor microenvironment and with the immune system culminating in the promotion of tumor growth and immune evasion.

## Conclusion

The role of microRNAs in the development and progression of lung cancer as well as other types of cancers is overwhelming; with several reports demonstrating the enormous impact microRNAs have on several cancer-associated processes.

In this review, we have elaborated on how microRNA-target interactions transcend beyond simple post-transcriptional regulation of oncogenes and/or tumor suppressor mRNAs to a more complex setting where they not only modulate networks and pathways, but also affect the tumor microenvironment, the epigenome and immune evasion. In lung cancer, their impact is very relevant, and to a large degree is deeply entrenched in several cascades, which impact lung cancer progression and metastasis. Inherently, microRNAs can target several molecules concurrently, and using this advantage together with the identification of the right molecule in the right context could have great potential, especially when used alongside other therapeutic modalities. Their involvement in several critical cancer associated processes makes them highly interesting molecules. Their effects transcend simple intracellular events, and are able to influence neighboring cells and even those at distant sites. Sufficient evidence indicates that they are significant modulators of our immune system which widens their scope as potential therapeutic agents.

Despite the tremendous amount of knowledge we have already on microRNAs, new publications keep coming out, describing yet other novel functions, making us marvel about the wide-reaching potential of these small molecules. In summary, microRNAs seem to be a very promising research target, however, the complexity of their actions makes keeping this promise very challenging.

## Abbreviations

CAF: Cancer associated fibroblasts
CTL: Cytotoxic T-cell
DNMT: DNA methyltransferase
EMT: Epithelial to mesenchymal transition
ECM: Extracellular matrix
HAT: Histone acetyltransferase
HDAC: Histone deacetylase
HMT: Histone methyltransferase
M-CSF: Macrophage colony stimulating factor
MVD: Microvessel density
MSC: Mesenchymal stem cells
NKC: Natural killer cells
NSCLC: Non-small cell lung cancer
TAM: Tumor associated macrophages
Tregs: Regulatory T-cells
